# Design of Online Music Education System Based on Artificial Intelligence and Multiuser Detection Algorithm

**DOI:** 10.1155/2022/9083436

**Published:** 2022-03-24

**Authors:** Hua Yan

**Affiliations:** Zhejiang Yuexiu University, Shaoxing, Zhejiang 312000, China

## Abstract

With the development of information technology, online music education has become a mainstream education method. Especially after the outbreak of COVID-19, music teachers have to teach through online. Therefore, an online music education system that can improve the quality of teaching is particularly important. Multiuser detection algorithms and artificial intelligence have important applications in many fields, and the field of music online education is no exception. This paper takes the music teaching of the music distance teaching unit as the goal and conducts sufficient research on the educational subjects such as teachers, students, and administrators. And with the help of the SCMA system multiuser detection algorithm and artificial intelligence technology, the system analysis and design method is used to analyze and design the music teaching function system. The system module involves basic information management, student music assignments, online courses, and other levels, providing an excellent educational system design example for music online education. The conclusion analysis shows that the music online education system based on SCMA system multiuser detection algorithm and artificial intelligence designed in this paper can significantly improve the audience's music learning efficiency and has obvious benefits to the student group.

## 1. Introduction

Most students believe that the teaching level of teachers determines the professional level of students to a certain extent. Under the traditional teaching mode, education is often led by the teacher. They choose the content of the course and the amount of work, and the teacher teaches and corrects homework. However, in the process of continuous in-depth research on education, people have found that student-centered education can often bring better results to education. About music, training can be divided into six links, such as analyzing the needs of training, formulating training plans according to different needs, preparing for training according to the plan, and evaluating and improving the content of the training after the implementation of the training plan. The process of music training demand analysis mainly analyzes the ability and level of the trainer, the current education level, and the current hot spots. Targeted training needs to be conducted in these areas. Therefore, in the process of music education, more and more attention is paid to the current knowledge and ability of the educator, instead of teaching knowledge in the traditional way and passively accepting music concepts. This is also in line with the basic elements of education in educational theory [1–3].

In the entire education industry, more and more attention is paid to the application of artificial intelligence technology. Artificial intelligence technology can be used to analyze customer consumption habits, make use of data support to provide a reference for decision-makers, and then carry out some targeted business activities [4]. Therefore, the author believes that the integration of artificial intelligence technology in the education industry can allow students to get more accurate knowledge mastery and other related knowledge and then carry out targeted training for the educated to improve the ability of the educated that will ultimately expand the connotation of education.

In this article, the author first studied the SCMA system and systematically understood the principles of the sender and receiver applications, as well as the key technologies applied in the system. For the receiving end of the SCMA system, as the number of users increases, the search space and the number of iterations will also increase, resulting in an increase in complexity [5, 6].

## 2. Related Work

Literature [7] proposed a new low-density sequence, which is conducive to solving the problems of CDMA technology. Literature [8] uses a new type of sparse spreading sequence. This method avoids the problem of the lack of orthogonal and approximately orthogonal code words. Literature [9] can separate users' information by using information transfer algorithms. When the available broadband transportation environment and service quality remain unchanged, the most important factor in the multiple access scheme is the number of users. In [10], in order to ensure that the performance of the spread spectrum code is still the same as that of a single user when most people use the spread spectrum code, the system capacity is expanded by using a low-density spread spectrum sequence and various technologies. The SCMA technology is formed on top of the LDS-MA technology, which can be applied to 5G mobile communications. Because of the rich and diverse technical version designs, the transceiver must know the codebook to be able to transmit signals, which improves security to a certain extent. For factor graphs, a check matrix can be selected, and the selected check matrix often has the characteristics of low density and parity. Because the multiple access mode is very special, the overload rate can be as high as 300%. At present, there have been some studies on the design of multibit constellations, but SCMA requires better power classification with optimal product distance numbers and multidimensional code words with high correlation. This helps simplify the detection and improve the performance of the system. As for the detector, since this technology was proposed late, the detection algorithm used is particularly rare. According to the iterative idea of literature [11], the MPA algorithm can be used to continuously approach the conditions. Although the current performance is very superior, the complexity of the algorithm is not certain because the number of iterations required is very large. As users increase, complexity will increase, and this increase exhibits exponential characteristics. Literature [12] because the current detection algorithm cannot meet the existing requirements, a new detection method is proposed. This method is used for the transmission of fixed and low-complexity messages on the uplink, which greatly reduces the complexity. Therefore, new low-complexity multiuser detection algorithms should be adopted. Literature [13] designed an attention-enhanced graph convolutional LSTM network for skeleton-based action recognition. Literature [14] designed a music-assisted teaching system based on artificial intelligence technology.

## 3. Theoretical Analysis of SCMA System Multiuser Detection Algorithm

### 3.1. SCMA Codebook Design

In SCMA technology, codebook design and multiuser detection technology are applied to enhance the efficiency of spectrum utilization. The introduction of a multidimensional constellation into the codebook design has significantly improved the system. The MPA detection technology also effectively controls the complexity of receiving, and it is closer to the characteristics of MAP during data detection and reception. The design technology and detection technology of the codebook can be introduced in detail below:

(1) $$\begin{array}{c} C*=\arg\underset{c\in C}{\min}{\left\|c\right\|}^{2}, \end{array}$$

where ‖*c*‖^2^ is the appropriate given design criterion and *C∗* is the definition and solution of this kind of multidimensional problem. According to the minimum value, the suboptimal solution of the problem is finally realized.

### 3.2. SUMIS: MPA Multiuser Detection Algorithm Model

The SUMIS and MPA algorithm can be divided into two processes. The first process is to calculate the posterior probability and send the code word based on the estimated result. The second stage is to perform interference, control, and multiuser detection on the obtained data. In the SCMA system structure, the receiving vector of the receiving antenna at the receiving end can be expressed as follows:

(2) $$\begin{array}{c} y=\sum_{j=1}^{J}H_{j}x_{j}+e=\sum_{j\in \Gamma_{n_{s}}}H_{j}x_{j}+\sum_{j\in \Gamma_{J-n_{s}}}H_{j}x_{j}+e\overset{\Delta }{=}\bar{H}\cdot \bar{x}+\tilde{H}\cdot \tilde{x}+e. \end{array}$$

A variety of segmentation and arrangement methods can be used to segment and arrange the user's sent code words. In this article, a similar model of the receiving end is defined as follows:

(3) $$\begin{array}{c} \bar{y}\overset{\Delta }{=}\bar{H}⊕\bar{x}+n. \end{array}$$

When the random variables are independent of each other, the sum of the random variables is similar to the Gaussian distribution. The variance is calculated as follows:

(4) $$\begin{array}{c} Q=\sum_{j\in \Gamma_{J-n_{s}}}H_{j}\Psi_{x_{j}}H_{j}^{H}+N_{0}I. \end{array}$$

The SCMA code word is sparse, and the covariance matrix of the transmitted symbol is as follows:

(5) $$\begin{array}{c} \Psi_{x_{j}}=V_{j}V_{j}^{H}\text{diag}\left(P_{j}\right). \end{array}$$

The transmit power of each dimension of the code word sent by the user is represented by *E* here. Therefore, the following model is an approximate model:

(6) $$\begin{array}{c} p\left(y|\bar{x}\right)=p\left(\bar{y}|\bar{x}\right)|{}_{\bar{y}=y}. \end{array}$$

By approximating *Y*, we can deduce

(7) $$\begin{array}{c} \;P\left(\bar{X}|y\right)\propto p\left(y|\bar{X}\right)\approx p\left(\bar{y}|\bar{X}\right)|{}_{\bar{y}=y}. \end{array}$$

By approximate marginalization, the posterior probability of code word *x* can satisfy

(8) $$\begin{array}{c} P\left(x_{j}|y\right)|{}_{\bar{y}=y}\propto \sum_{\bar{X}:X_{j}=X}p\left(\bar{y}|\bar{x}\right)|{}_{\bar{y}=y},p\left(\bar{y}|\bar{x}\right)|{}_{\bar{y}=y}=\frac{1}{\pi^{K}\left|Q\right|}\exp\left(-{\left\|\bar{y}-\bar{H}\Theta \bar{X}\right\|}_{Q}^{2}\right). \end{array}$$

From the above formula, the required prior probability can be obtained, namely

(9) $$\begin{array}{c} \sum_{m=1}^{M}P\left(x_{j}=s_{j,m}|\bar{y}\right)=1. \end{array}$$

Then

(10) $$\begin{array}{c} \lambda_{j,m}\overset{\Delta }{=}\log\left(\frac{P\left(x_{j}=s_{j,m}|\bar{y}\right)}{P\left(x_{j}=s_{j,1}|\bar{y}\right)}\right)|{}_{\bar{y}=y}=\log\left(\frac{\sum_{\bar{x}:x_{j}=s_{j,m}}p\left(\bar{y}|\bar{x}\right)}{\sum_{\bar{x}:x_{j}=s_{j,1}}p\left(\bar{y}|\bar{x}\right)}\right)|{}_{\bar{y}=y}\\ =\log\left(\frac{\sum_{\bar{x}:x_{j}=s_{j,m}}\exp\left(-{\left\|\bar{y}-\bar{H}\Theta \bar{x}\right\|}_{Q}^{2}\right)}{\sum_{\bar{x}:x_{j}=s_{j,1}}\exp\left(-{\left\|\bar{y}-\bar{H}\Theta \bar{x}\right\|}_{Q}^{2}\right)}\right). \end{array}$$

The relationship between the probabilities is as follows:

(11) $$\begin{array}{c} P\left(x_{j}=s_{j,m}|\bar{y}\right)|{}_{\bar{y}=y}=P\left(x_{j}=s_{j,1}|\bar{y}\right)|{}_{\bar{y}=y}e^{\lambda_{j,m}}. \end{array}$$

The above formula can be brought into

(12) $$\begin{array}{c} P\left(x_{j}=s_{j,1}|\bar{y}\right)|{}_{\bar{y}=y}=\frac{1}{\sum_{m=1}^{M}e^{\lambda_{j,m}}}. \end{array}$$

It can be derived from the above formula that the received signal *y* is used to determine *x*, and the conditional probability of *s* plus is

(13) $$\begin{array}{c} P\left(x_{j}=s_{j,1}|\bar{y}\right)|{}_{\bar{y}=y}=\frac{e^{\lambda_{j,m}}}{\sum_{m=1}^{M}e^{\lambda_{j,m}}}. \end{array}$$

In order to eliminate interference, the expectation of *x* needs to be required to eliminate interference.

(14) $$\begin{array}{c} E\left\{x_{j}|\bar{y}\right\}\approx \sum_{m=1}^{M}s_{j,m}P\left(x_{j}=s_{j,\text{m}}|\bar{y}\right)|{}_{\bar{y}=y}. \end{array}$$

By sending code words and splitting the channel matrix to reduce the complexity, the stability of the value is basically guaranteed, and the hardware can be realized by calculating a fixed number of points. In order to find the expectations of other user code words in *X*, it can be suppressed by the following formula:

(15) $$\begin{array}{c} y\prime \overset{\Delta }{=}y-\sum_{j\in \Gamma_{J-n_{s}}}H_{j}E\left\{x_{j}|\bar{y}\right\}\approx \bar{H}\Theta \bar{x}+n^{\prime }. \end{array}$$

Define the interference in the above formula as follows:

(16) $$\begin{array}{c} n\prime \overset{\Delta }{=}\tilde{H}\Theta \left(\tilde{x}-E\left\{\tilde{x}|y\right\}\right)+e. \end{array}$$

Similar to the previous interference, by the central limit theorem, its variance is

(17) $$\begin{array}{c} Q\prime =\sum_{j\in \Gamma_{J-n_{s}}}H_{j}\Phi_{x_{j}-E\left\{x_{j}|\bar{y}\right\}}H_{j}^{H}+N_{0}I. \end{array}$$

For interference *i* independent of the received signal *Y*, we can get:

(18) $$\begin{array}{c} \tilde{\Phi }=E\left\{\tilde{x}\cdot {\tilde{x}}^{H}|y\right\}-E\left\{\tilde{x}|y\right\}\cdot E{\left\{\tilde{x}|y\right\}}^{H}. \end{array}$$

After removing the conditional mean of interference *i*, a new matrix can be obtained. We use the MPA algorithm to detect the new factor matrix.

### 3.3. Research on Existing Detection Algorithm of SCMA System

The principle of SCMA in multiuser detection is basically the same as the detection methods in other systems. When performing multiuser differentiation, the maximum posterior probability of each user's signal sent is used to complete the detection target. The MAP detection method can be used to calculate the maximum posterior probability and determine the sequence value of the detection. The estimated results are as follows:

(19) $$\begin{array}{c} x_{j}^{n}\prime =\arg\underset{a\in X}{\max}\sum_{x\in X^{N}\omega_{j}=a}p\left(x|y\right). \end{array}$$

According to the above formula, the posterior probability of the summation term can be realized by the conversion.

(20) $$\begin{array}{c} p\left(x|y\right)\propto p\left(y|x\right)P\left(x\right). \end{array}$$

The noise vector and the sending vector are independent of each other, and the noise vector also shows the same distribution law. There is a significant feature in SCMA technology that is the sparse factor graph. According to this feature and the observation value of each chip, the formula can be further changed as follows:

(21) $$\begin{array}{c} p\left(y_{k}|x\right)=p\left(y_{k}{|x}^{\left[a\right]}\right)=M_{k}\left(x\right). \end{array}$$

The MAP algorithm can be further optimized. After likelihood detection, it is estimated based on the symbol of a user on the chip:

(22) $$\begin{array}{c} x_{j}^{n}\prime =\arg\underset{a\in X^{N}}{\max}\prod_{k=1}^{K}M_{k}\left(x\right). \end{array}$$

Then the local channel observation value on the *K*-th antenna can be calculated. The author got inspiration from the maximum sum-product algorithm in the LDPC code decoding problem. The author believes that the problem of MAP detection can be converted by sparse information and become an MPF problem. After MPF processing, the corresponding factor graph can be used in MPA.

## 4. Design and Test of Music Online Education System Based on Mobile Platform

### 4.1. System Outline Design

In order to make the system more stable, the system can be divided into three levels to maintain and expand the system.

1. Data layer: The data layer can provide an interface for the system to access data and can perform a series of operations on the data on the database platform. The data types of the system include not only objects in the database but also user passwords. Use JDBC to operate the database, such as querying the data in the database and uploading relevant information to the database, and update the data for the first time. The system database also contains basic information about students, as well as the relevant information and question bank of the students' performance.
2. Business logic layer: In this layer, the formulation of business rules can be realized, and the business logic of the system can be defined at the same time. Generally, the storage of business logic definitions can be realized in two ways [15]. One is an XML file, and the other is a database table. The information setting can be completed in the reading and writing of the data table record, and the logic can be set and read in the JavaBean to provide information on the processing result.
3. Functional performance: The functional performance layer can connect users and the system. When the user operating system inputs data or selects options, it can be submitted to the server by the system. Next, we can see the calculation process on the server, including not only the prompts of the operation results but also the data query results and so on [16]. The functional authority layer contains a variety of operation pages, such as basic information management, assignment of homework, practice management results, communication facilities management, and so on. The hierarchical design makes the system more expandable. The system can change the business logic at any time according to the needs of customers, and the change process is very simple. Expanding in the business layer or making changes to the business from the original data can eliminate the need to adjust business logic or modify the front-end business, greatly reducing maintenance costs [17]. The physical structure of the system is connected through the physical network of the system and is associated with user terminals. Each user can connect to the mobile communication network through a mobile phone to inquire about information or access the background through the desktop system. Students can complete music learning online through mobile phones (Figure 1).

### 4.2. System Detailed Design

Through the above analysis, we can find that user information management includes not only query and statistics but also some basic operations such as maintenance. Maintenance actually allows users to add, modify, or delete operations. Users can query the information they want by entering keywords, which is user query [18]. The user statistics is that the user classifies the user information in the database by entering the conditions that they want to count.  Figure 2 shows the design of the user information management class. Among the user information management category, the database connection is realized through the DB class; operations such as modification and deletion of information in the database, or addition, can be realized through the data set; usually users can be added or removed or deleted and modified for statistical work. There are also fixed categories for user information query operations and user statistics operations. Different categories can meet the different needs of customers.

The music job management module includes not only music job query but also a series of operations related to it, such as uploading music job and maintenance. The design of the music homework management class is shown in Figure 3. In this module, resource files are designed to facilitate educators to manage music homework. In this module, it is very convenient to query, add, save, and delete operations. Music assignments contain different types, such as audio, video, and text data, so the way they open the page should not be the same. Files can be displayed through showfile and uploaded through upload.

In the classification design, resources should be taken as entities. You must first specify the number of the resource. You can upload the resource file, check whether it is not displayed, and delete the content contained in the resource file. It can be realized through display and control. Students can complete music exercises through mobile phones [19]. In order to make the exercises more effective, the system can make sounds through mobile phones, including accompaniment questions and demonstrations of famous works. In order to meet the needs of students and parents, an extended grade import class is also set. Information about students is classified and recorded. Maintain students' practice operations through works, use student ID to represent students, and use work Id to represent students' works [20]. Use del, add, save, and so on to complete the processing, addition, and storage of works, respectively, and query, import, and delete through search, import, and del, respectively. Each part has a corresponding indicator.

The score contains not only the basic score of the student but also the student's practice score. You can click on the student logo to get the details of the practice score. In the student classification, you can get the student's practice questions and practice results. Some methods of using other attributes of the classification have been described before and will not be described in detail in this paragraph.

Online classroom not only realizes the online interaction between students and teachers but also includes some forms of online questioning, browsing resources, and homework assignments [21]. Online classes meet the needs of students to set goals and achieve them. After setting goals, students can enter the system for testing and learning at any time. During the learning process, you can use the tools provided under the module, take notes, leave your thoughts, and raise questions, and you can discuss them in future learning. After the students' study, the system will automatically record the results of this time for teachers to conduct subsequent assessments.  Figure 4 shows the design of the online classroom. This module involves the online classroom learning log, learning reflection, and student information management [22]. In online classrooms, when music homework is needed, teachers can use resources to get the students' homework, and students can also get the latest assignments through resources, start self-learning, and record the learning process through the learning logo, such as the start of learning time and time to complete the job.

At this stage, the music teaching system has been widely adopted. Some teaching information and dynamics can be released through the platform. The system can send the dynamics released by the teacher to each student's mobile phone in the form of a push. According to past experience, the system information and some teaching notices are actually similar. They have two parts: one is basic information, and the other is attachment information. When the system is managing this information, it only needs to design a big category to complete the notification and maintenance of related information.

The design process of the system function can be understood through class design.  Figure 4 shows the class design of information notification. Publicity includes information and communication information, and basic information can be added or modified in public information. You can get the information you want through get publicity for and display it through the system. Adding, deleting, saving, and querying company information can all be implemented in this category. After the complete information is released, the information can be released in a timely manner, the receiver can inquire, browse, and save in time, and the notifier and publisher of the message can also delete the information in time [23]. Notice is a category under the information announcement category. On the basis of the release of inherited information, the above operations are performed on the daily notification information. Through file manager, you can perform operations on attached files, such as querying information, browsing information, uploading information, and so on.

### 4.3. System Database Design

On the basis of system analysis and system design, understand the function of the system. A system must have a database, so it is necessary to design a complete system database. In this paragraph, we understand the design of the database by establishing a conceptual model of the system database and describing the physical structure [24]. There are three parts in the construction of the database. In this part, the conceptual model diagram of the database can clearly describe the design philosophy and logic of the system. The core table is used when describing the physical design of the database. In the physical design process of the database, the database table design is a very important part. Only when the structure of the data table is complete can the database physical design be better [25]. The physical structure is described through tables.

Attachment information, as the name implies, is an attachment that explains or collects the main information. The information in the attachment is often stored in the form of a file in the system. The title, category, and address of the stored document can be found in the attachment information table.

Some information on daily notifications can be found in the daily notification information table, including basic information of notifications, information to be browsed, and so on.

The homework public information table can store the homework information released by the teacher in the table in a timely manner. The table contains basic function information, homework released by the teacher, browsing information, and so on.

### 4.4. System Development Environment

System development is carried out on Windows7; the integrated development environment is MyEclipse6.0; the development language used is Java; and the web client uses HTML5 + JavaScript. The version used by the client is above Android 4.0, and ADTBundle is used for client development under MyEclipse. The details are shown in Table 1.

### 4.5. System Test and Result Analysis

A series of tests were carried out before the system was put into use. After simulating the classroom process of students and teachers, the author believes that the two roles of student and teacher can maintain the music homework and can also check the usage of homework [26]. No problems were encountered during the process. In order to avoid accidentally touching the deletion indicator, the system will pop up a dialog box to give reminders when deleting data to ensure data security (Table 2).

Table 3 is the online classroom module function test table. By taking tests, it can be judged whether students can complete a series of operations with the system.

There are two main tests for system performance: one is the stress test, and the other is the failure recovery test. Several typical services were selected during the test, and they were run on LoadRunner after completing the settings and writing scripts [27]. Investigate the performance response of the system by analyzing the operating results. During the experiment, multiple virtual users were established. Below, the author will describe the testing process from two levels: stress testing and recovery testing.

#### 4.5.1. Stress Test

During the test, select several commonly used system functions, simulate the number of users, and set the number of virtual users to 4,000, 5,000, and 6,000 according to the number of people in each department in the system and the number of people in the application system. Visit under different test conditions. View the results of the stress test through load runner. The result of the test is actually the response time. It means when the system receives and returns the result after the user submits the request [28]. Even if the number of users reaches 6,000, the response time of the system will not exceed three seconds, so the author thinks that the response time can meet the requirements of the system, and people often query some more complex data. After testing this aspect, the author believes that the response time of the system cannot exceed 9 seconds when performing complex data services.

#### 4.5.2. Recovery Test

The recovery test is how long it takes to restore the original state for normal access when the system has a problem. Generally speaking, the abnormality of the system service is only discovered when the user accesses it. The server shows that when many users visit together, they need to process user requests in batches.  Table 4 shows the system performance test.

## 5. The Role of Them in Promoting Online Music Teaching

### 5.1. Strengthening the Teaching Atmosphere

Online education often cannot make people immersive, mainly because online education is not personalized and there is less interaction between teachers and students. Applying big data in online education can understand students' learning habits, accumulate some data in the learning process of students, and analyze students' mastery of courses. Students can ask questions to teachers online, and students can also communicate with each other. This will make it easier for students to devote themselves to teaching and greatly improve their learning effects. Some technologies in artificial intelligence, such as voice recognition and face recognition, can help students and teachers interact in the classroom.

First of all, big data can clearly record the time for students to log in to their account and the time for students to learn knowledge points, the number of times they browse videos, the probability of answering class exercises, and the correct rate of exercises [29]. Teachers can use these data to analyze and compare to master students. The level of understanding of knowledge points can find out the gap between the students' current learning situation and their goals. Through the following education process, students' ability to grasp knowledge can be improved, and this gap can be shortened to achieve the goal of education. Teachers can also adjust the teaching plan based on the feedback of students. After mastering the needs of students, they can achieve targeted and personalized education and truly strengthen the pertinence of teaching.

Secondly, the questions that students have during the learning process can be recorded by big data after they are entered into the background [30–32]. Teachers can concentrate on answering where most students have questions. In this way, the shortcomings in traditional learning are greatly compensated, and teachers can answer students' questions at any time. Students who have the same questions can discuss with each other and interact with each other through expert answers or other forms to enhance the teaching experience.

Finally, the use of them can grasp the learning status of students, enhance students' experience, and help achieve personalized teaching. Through facial recognition technology, teachers can view students' expressions in time and learn about students' knowledge points through student expressions [33]. After receiving information of students' performance, the teacher can adjust the teaching plan and methods in time to realize personalized teaching. Speech recognition and language understanding technologies under big data can make online education closer to real education. In the process of online course education, students can deepen their understanding of learning content through questions or discussions. Teachers can ask students questions through big data voice recognition. After the voice input recognition is used to provide feedback to their own answers to the students, this will truly achieve the same interaction as classroom education.

In summary, they can give great help for education so that teachers have a more on-site teaching sense, and students can be more immersive [34]. Teachers can accurately judge the level of mastery of each student. Use facial expressions to judge whether students have questions about a certain problem. For every student, the teacher can give targeted guidance on areas that he has questions about. In the near future, when big data and artificial technology are used proficiently, online education can also bring students a good course experience like on-site teaching, making students more willing to accept online education for learning.

### 5.2. Reshaping the Online Teaching System

There are also some shortcomings in online education. Online education pays more attention to fragmented learning. Students learn a lot of content, and it is difficult to choose courses that suit their level. And if big data and artificial intelligence are used in the teaching process, science and technology can be used to analyze students' learning interests and learning habits and record students' mastery of a certain knowledge point during the learning process. Analyzing the learning information of students can accurately grasp the needs of students [35]. The system can match the most suitable courses for students according to their current learning ability and their hobbies. Students not only need not worry about choosing courses but can also upgrade their knowledge [36]. So, after long-term development, students' satisfaction with courses will increase, and society will recognize online education more [37–40].

### 5.3. Improving the Construction of the Curriculum System

Online education often has the problem of a low completion rate. This is mainly because students lack self-discipline. Teachers cannot judge whether students are in a class by seeing students in front of computers. Students do not have a certain interest in the course, and their attention is often placed on the things they are interested in. Therefore, although most of the trading platforms have added functions such as sign-in and face recognition to urge students to study and complete course tasks every day. But these measures can only remain effective for a short time. Through the data, we can find that the success rate of the courses that students are interested in is often very high. This is because students think that when learning the content of interest, time often flies quickly, which has a multiplier effect. For example, elementary and middle school students do not have a high degree of mastery of subject knowledge and learning logic, but once games are involved, what they know is very comprehensive, and they are well-founded when discussing. Therefore, we can think that students have strong logical thinking abilities and can do better in learning. Big data and artificial intelligence can be used to determine students' behaviors and hobbies, match students with more interesting courses, and combine the topics of interest with books, and the courses will become more attractive. Students will participate in learning with interest so that the completion rate of the course will be greatly improved.

## 6. Conclusion

The SCMA system multiuser detection algorithm and artificial intelligence play a role in promoting the development of all industries. The integration of artificial intelligence into the SCMA system multiuser detection algorithm accelerates the creation of value and makes a positive impact on promoting the sustainable development of future industries.

At present, online music education, combining the SCMA system multiuser detection algorithm with artificial intelligence, is a future development trend. The Internet and educational technology are essential for online music education. The development of artificial intelligence can give people a new understanding of online education. It means online education may become more attractive and will be generally recognized by people. In this research, the goal is set as the music teaching of music distance teaching units, and the subjects of education such as teachers, students, and administrators have been fully studied. System analysis and design for music teaching functions. The system modules involve various levels, such as basic information management, student music homework, online courses, and so on. The use of this system provides an excellent education system for music online education.

## Figures and Tables

**Figure 1:** System physical structure diagram.

**Figure 2:** User information management design.

**Figure 3:** Music assignment management design.

**Figure 4:** Information notification class design.

**Table 1:** System environment configuration.

Software	Configure
Development language	Java, HTML5 + JavaScript
Basic software platform	MyEclipse6.0
Tools	ADTBundle
Operating system	Android 4.0

**Table 2:** Function test table of music job management module.

Serial number	Test items	Testing method	Test results
1	Music job information input	Enter the entry interface, enter some illegal data, test whether it can be saved, record fewer required items, and test whether it can be saved	Adopt
2	Music assignment information modification	Select a piece of music assignment information, modify a piece of information, and test whether it can be saved after modification	Adopt
3	Music assignment information deletion	Whether the music job information can be deleted correctly, test whether there is a prompt message before deleting it	Adopt
4	Music assignment letter upload	Complete the attachment upload by selecting the music job	Adopt

**Table 3:** Online classroom module function test form.

Serial number	Test items	Testing method	Test results
1	Learning log	Students choose some courseware resources on the Internet, complete online playback, and test whether the system records their learning logs	Adopt
2	Music homework browsing	Can students complete the online browsing of music homework by querying some keywords?	Adopt
3	Online classroom questions	Test whether you can complete online question consultation after passing the online classroom module	Adopt
4	Teacher online classroom solution	Pass the teacher role test whether to pass the selection question and answer the question	Adopt

**Table 4:** System performance test.

Test items	System stress test			
Test index	Under the condition of simultaneous access by multiple concurrent users			
Test conditions	The test script has been compiled; load runner has been debugged			
Step	Number of virtual users established	Number of users expected to pass	Number of users actually passed	Regression testing
1	100	100	100	1
2	500	500	500	2
3	1,000	1,000	1,000	3
4	2,000	2,000	2,000	4
5	3,000	3,000	3,000	5
6	5,000	5,000	5,000	6

## Data Availability

The data sets used and/or analyzed during the current study are available from the corresponding author on reasonable request.
